# Cell and tissue tropism of enterovirus 71 and other enteroviruses infections

**DOI:** 10.1186/1423-0127-21-18

**Published:** 2014-03-07

**Authors:** Jing-Yi Lin, Shin-Ru Shih

**Affiliations:** 1 School of Medical Laboratory Science and Biotechnology, College of Medical Science and Technology, Taipei Medical University, Taipei, Taiwan; 2 Research Center for Emerging Viral Infections, Chang Gung University, Tao-Yuan, Taiwan; 3 Department of Medical Biotechnology and Laboratory Science, Chang Gung University, Tao-Yuan, Taiwan; 4 Clinical Virology Laboratory, Chang Gung Memorial Hospital, Tao-Yuan, Taiwan

## Abstract

Enterovirus 71 (EV71) is a member of *Picornaviridae* that causes mild and self-limiting hand, foot, and mouth disease (HFMD). However, EV71 infections can progress to polio-like paralysis, neurogenic pulmonary edema, and fatal encephalitis in infants and young children. Large EV71 outbreaks have been reported in Taiwan, China, Japan, Malaysia, Singapore, and Australia. This virus is considered a critical emerging public health threat. EV71 is an important crucial neurotropic enterovirus for which there is currently no effective antiviral drug or vaccine. The mechanism by which EV71 causes severe central nervous system complications remains unclear. The interaction between the virus and the host is vital for viral replication, virulence, and pathogenicity. SCARB2 or PSGL-1 receptor binding is the first step in the development of viral infections, and viral factors (e.g., 5′ UTR, VP1, 3C, 3D, 3′ UTR), host factors and environments (e.g., ITAFs, type I IFN) are also involved in viral infections. The tissue tropism and pathogenesis of viruses are determined by a combination of several factors. This review article provides a summary of host and virus factors affecting cell and tissue tropism and the pathogenesis of enteroviruses.

## Review

### Introduction

Enterovirus 71 (EV71), a member of the family *Picornaviridae*, poses a persistent global public health threat. EV71 infections typically cause hand, foot, and mouth disease (HFMD) or herpangina; however, EV71 has also been implicated as the etiological agent in several large-scale outbreaks of severe neurological complications in children worldwide [1]. In recent years, an increase in EV71 activity has been noted throughout the Asia-Pacific region [2-6]. Severe neurological complications, including brainstem encephalitis, meningitis, poliomyelitis-like paralysis, and even death have occurred in this region. In 1998, an EV71 epidemic occurred in Taiwan, with the virus infecting over 120000 people and killing 78 children. Numerous small-scale EV71 epidemics have also occurred since 1998 in Taiwan [2].

EV71 is a positive-stranded RNA virus [7]. This viral RNA has a small protein named VPg covalently attached to its 5′ end and is polyadenylated at its 3′ terminus. The genomic RNA is approximately 7500 nucleotides long. The 5′ untranslated region (5′ UTR) is 745 nucleotides long and highly structured, containing a cloverleaf-like structure that is integral for viral RNA synthesis and an internal ribosomal entry site (IRES) that is critical for the direction of viral mRNA translation. The cloverleaf-like structure at the 5′ end of this region is a multifunctional, *cis*-acting replication element that interacts with viral and cellular proteins to form a ribonucleoprotein complex. The approximately 450-nt IRES in the 5′ UTR mediates the initiation of picornavirus translation. When the 40S ribosomal subunit recognizes a sequence, RNA structure, or ribonucleoprotein complex within the IRES, initiation occurs at the authentic start codon. It has been reported that cellular proteins (such as poly(C)-binding protein 1 (PCBP1), poly(C)-binding protein 2 (PCBP2), polypyrimidine tract-binding protein (PTB), heterogeneous nuclear ribonucleoprotein A1 (hnRNP A1), heterogeneous nuclear ribonucleoprotein K (hnRNP K), La, upstream of N-ras (Unr), far upstream element binding protein 1 (FBP1), and far upstream element binding protein 2 (FBP2)) associate with the picornaviral 5′ UTR and participate in either viral RNA replication or viral IRES activity, or both [8-14]. The viral RNA encodes a single large polyprotein, which undergoes several self-processing events that are mediated by virus-encoded proteases (2A and 3C) to produce mature viral proteins (including 11 mature proteins and numerous partially processed products, depending on the virus). Four of these proteins (VP1-VP4) constitute the virus capsid, and the others participate in viral replication [15].

Pathogenesis is a multistep process: the virus-receptor interaction is the first step to initiating infection and the development of a disease is influenced by the intracellular milieu; induced cell functions, such as the capacity of the host to develop an effective immune response; the speed of virus replication; cytopathogenicity; and the spread of infection within and between tissues or organs, which might or might not depend on the presence of specific or different cellular receptors. This article reviews viral and host factors involved in the cell and tissue tropism of enteroviruses.

### Viral factors contribute to cell and tissue tropism

EV71 serotypes are divided into 3 major genetic lineages: lineage A for which the prototype is the BrCr strain, and lineages B and C, which are further subdivided into subgenogroups B1 to B5 and C1 to C5 [3,16]. Previous animal studies have shown that a mouse virulent strain of human EV71 belonging to subgenogroup B3 by serial passage is present in newborn BALB/c mice (MP-26 M). This virus strain expressing the VP1-G145E mutation increases viral growth and virulence in mice [17]. In the subgenogroup-B5 mouse-virulent EV71 strain, viruses expressing VP1-K244E mutation are critical genetic determinants of virulence [18]. Previous studies have reported that the C1 subgenogroup is rarely the cause of central nervous system (CNS) infections [3,4]; however, modifying a key mutation (Q145E) into capsid protein VP1 of the subgenogroup-C4 strain of EV71 generates a mouse-virulent EV71 strain [19].

Numerous studies have indicated that the 5′ UTR and 3′ UTR of enteroviruses exert a considerable influence on tissue tropism, neurovirulence, and viral pathogenesis [20-23]. Nucleotides 480, 481, and 472 in the 5′ UTR of PV are cited as neurovirulent determinants of PV1, 2, and 3 [24-26]. Stem-loop II within the 5′ UTR of CVB1 and CVB3 determines the cardiovirulence phenotype [27]. In addition, nucleotide C158 in stem-loop II of the 5′ UTR of unadapted isolated EV71 strain 237 contributes to virulence in mice [28].

Although previous studies in which animal models were used have succeeded in identifying genetic modifications that attenuate the virulence of enteroviruses, including coxsackieviruses, poliovirus, and EV71 [29-33], attempts to understand the underlying mechanism of virulence attenuation and the cell or tissue tropism of pathogenesis have not been assured.

Kok et al. reported that the modification of EV71 UTRs (5′ UTR and 3′ UTR) impairs growth in a cell-specific manner [34]. Replacing the entire EV71 5′ UTR with that of human rhinovirus 2 (HRV2) resulted in a small reduction in growth efficiency in cells of both nonneuronal (rhabdomyosarcoma; RD) and neuronal (SH-SY5Y) origin because of reduced translation efficiency. However, introducing a 17-nucleotide deletion into the proximal region of the 3′ UTR markedly reduced the growth of EV71-HRV2 in SH-SY5Y cells [34].

Cordey’s group analyzed the genome of EV71 from various sites of infection in an immunocompromised host with disseminated disease. In vitro reverse genetics experiments in various EV71 lineages and in silico modeling data showed that the VP1 BC loop region of EV71 (L97R) plays a critical role in cell tropism independent of the EV71 lineage and, thus, might have contributed to dissemination and neurotropism in the immunocompromised patient [35].

### Host factors modulate cell and tissue tropism

In addition to viral factors, several host factors are also involved in the cell and tissue tropism of enteroviruses.

### Receptors are the first step of viral infection

Infection of cells by a cell-free virus and virus spread from cell to cell are different processes that might depend on the presence of different cellular surface molecules. In infected organs, cell-to-cell spread contributes substantially to the pathogenesis of a viral disease. When enteroviruses infect humans, they target numerous organs, causing gastrointestinal, myocardial, respiratory, and CNS diseases. Virus infection initiates after the viruses bind to a receptor on the cell surface; cellular receptors for viruses have been considered the primary determinants of cell and tissue tropism and pathogenicity. Recently, human scavenger receptor class B member 2 (hSCARB2) and P-selectin glycoprotein ligand-1 (PSGL-1) have been identified as receptors for EV71 [36,37]. In addition, EV71 uses SA-linked glycans as receptors for infection [38].

hSCARB2, which was originally identified as an EV71 receptor on RD cells, is expressed on a broad variety of cell types. Scavenger receptor class B, member 2 (also known as lysosomal integral membrane protein II, LGP85, and CD36b-like-2) is composed of 478 amino acids and belongs to the CD36 family. hSCARB2 is one of the most abundant proteins in the lysosomal membrane and participates in membrane transportation and the reorganization of the endosomal/lysosomal compartment. Several studies have suggested that hSCARB2 plays critical roles in efficient EV71 infection and the development of disease in humans [37,39]. EV71 binds to SCARB2 through a canyon of VP1 around residue Gln-172 for virus infection, and the entire exon 4 of SCARB2 is responsible for the interaction with the VP1 protein of EV71 [39,40]. In addition, Coxsackievirus A14 (CVA14) and Coxsackievirus A16 (CVA16), which are also major causative agents of HFMD, also use hSCARB2 as a receptor [37,41]. Coxsackievirus A7 (CVA7), which is occasionally associated with neurological diseases as well as EV71, also uses hSCARB2 for infection [41].

Enteroviruses must escape host immune system defenses to reach the CNS, and can cross the blood–brain barrier and become disseminated to the CNS from the bloodstream, infected leukocytes, or neural cells [42]. For poliovirus, CNS invasion is thought to occur through either the disruption of the blood–brain barrier or retrograde axonal transport [43]. In contrast, PSGL-1, which was first identified as an EV71 receptor on Jurkat T cells, is primarily expressed on leukocytes, where it mediates interaction with selectins and thus serves a crucial function in inflammatory processes [36]. Some EV71 strains bind to PSGL-1 and infect immune cells, but others do not. Nishimura et al. observed that EV71 binds to the PSGL-1 N-terminus, and that binding depends on tyrosine sulfation of the N-terminus [44]. They also observed that a single amino acid, residue 145 of the viral capsid protein (VP1-145), determines whether a virus binds to PSGL-1, and that it functions by influencing the orientation of a nearby lysine residue (VP1-244) on the virus surface. They proposed that VP1-145 controls virus tropism by changing the accessibility of the positively-charged lysine side chain of VP1-244 to the negatively charged, sulfated N-terminus of PSGL-1. These results shed new light on virus-receptor interaction and EV71 tropism for PSGL-1-expressing leukocytes [45].

PSGL-1 is expressed mainly on leukocytes, but SCARB2 is widely expressed on various cell types, including neurons in the CNS. Moreover, unlike PSGL-1, SCARB2 can be used by most EV71 strains as an entry receptor [36,37]. Previous studies have reported that EV71 enters host cells through a mediated pH- and clathrin-dependent endocytosis pathway [46]. In addition, studies have reported that, to evaluate the role of SCARB2 and PSGL-1 during uncoating, the step of uncoating EV71 requires both SCARB2 and an acidic environment that forms after the virus-receptor complex is internalized into endosomes. However, this result was not observed in PSGL-1 [40,47]. Therefore, SCARB2 is capable of viral binding, viral internalization, and viral uncoating and greatly contributes to the early steps of EV71 infection [47].

### Other host factors

The replication of many viruses is restricted to certain cells and tissues in the host. This tissue tropism results in a distinct disease pattern unique to each virus. Because virus infection initiates after viruses bind to a receptor on the cell surface, cellular receptors for viruses have been considered the primary determinants of tissue tropism. However, after identifying receptors for numerous viruses, it became apparent that receptor distribution in the host is wider than that in the virus replication sites [48]. This indicates that virus tropism might be determined by factors other than the virus receptor.

### Internal ribosomal entry site transactivating factors (ITAFs) are involved in viral translation

The viral translation of enterovirus is IRES-dependent. IRES-mediated initiation might require both canonical initiation factors and IRES transactivating factors (ITAFs) that are not involved in cap-mediated initiation. ITAFs are cellular proteins that are not involved in normal cap-dependent translation but facilitate cap-independent translation. Different viral IRESs have different ITAF requirements, although several requirements are shared. ITAFs might serve as IRES chaperones, binding to RNA across multiple domains and stabilizing the entire IRES in a configuration that is appropriate for binding canonical translation factors, and ultimately ribosomes for translation. The ITAFs involved in enteroviruses replication and translation include PTB, nPTB, DRBP76, PCBP1, PCBP2, unr, La, hnRNP A1, hnRNP K, FBP1, and FBP2 [8-14,49]. However, some cellular factors, because of their cell and organ-specific distribution, might determine viral translation, propagation, virulence, and pathogenesis.

Mutations critical for the CNS attenuation of the Sabin vaccine strains of poliovirus are located within the viral IRES. The major determinant of neuroattenuation is a single-point mutation located within the viral IRES at nt 480, 481, or 472 in the cases of Sabin type 1 (Sabin1), Sabin2, and Sabin3, respectively [24-26]. A previous study showed that PTB and nPTB bind to a site directly adjacent to the nt 472 attenuating mutation, and binding at this site was less efficient on the Sabin3 IRES than on the PV3 IRES [23]. Translation mediated by the PV3 and Sabin3 IRESs in neurons of a chicken embryo spinal cord demonstrated a translation deficit for the Sabin3 IRES that could be rescued by increasing PTB expression in the CNS [23]. These data suggest that the low levels of PTB available in the CNS, as well as the reduced binding of PTB on the Sabin3 IRES, leads to its CNS-specific attenuation. Therefore, variable IRES *trans* activity of PTB and its neural isoform nPTB have been implicated in the neuroattenuation phenotype of the Sabin3 strain [23].

Some investigations have shown that doubled-stranded RNA-binding protein 76 (DRBP76) is associated with, and specifically repressed, the HRV2 IRES in neuronal but not in non-neuronal cells [49,50]. DRBP76 contains 2 dsRNA-binding motifs and is almost identical to M-phase phosphoprotein 4, NF90, translation control protein 80 (TCP80), and NF associated with dsRNA-1 (designated NFAR-1). Moreover, DRBP76 depletion in neuronal cells enhances rhinovirus IRES-driven translation and virus propagation [50].

### Interferon response controls tissue tropism and pathogenesis

Picornaviruses are sensitive to IFNs, which play a central role in the innate immune antiviral response. The alpha/beta interferon (IFN-α/β) response controls tissue tropism and the pathogenicity of poliovirus and coxsackievirus B3 (CVB3) [51,52]. AG129 mice lack alpha/beta interferon and IFN-γ receptor genes and were initially generated to study the in vivo antiviral effects of IFN-α/β and IFN-γ [53]. When AG129 mice were infected with a non-mouse-adapted strain of EV71 (5865/SIN/00009), the virus exhibited neurotropism and caused neurological damage that was likely responsible for the limb paralysis observed in the infected AG129 mice [54].

Enteroviruses may enter the CNS through the blood–brain barrier (BBB) or through axonal transport from the periphery. The host systemic adaptive and CNS innate immune systems express pattern-recognition receptors (PRRs) (endosomal Toll-like receptors (TLRs), cytoplasmic retinoic acid-inducible gene 1 (RIG-1), and melanoma differentiation-associated gene 5 (MDA-5)), which detect viral nucleic acids and initiate host antiviral responses. MDA-5 is a crucial factor for EV71 RNA-activated type I IFN expression [55]. However, EV71 inhibits the type I IFN response mediated by RIG-1 and TLR3, and this process involves the 3C viral protease that cleaves interferon regulatory factor 7 (IRF7) [56-58]. In addition, EV71 viral 3C protease inhibits the host cell antivirus type I IFN response promoting virus replication in mice [59].

### Roles of microRNAs in the interaction network between virus and host

In addition to host proteins and viral genome diversity, some small RNAs have been reported to be involved in regulating viral replication and translation in viral life cycles [60-63]. MicroRNAs (miRNAs) are a recently discovered class of RNAs with the function of posttranscriptional gene expression regulation. It has been demonstrated that miRNAs play crucial roles in the complex interaction network between a virus and a host [64]. miRNA expression is tissue dependent and the abundance of a particular miRNA might present a clue regarding whether it functions in the tissue [65]. Group B coxsackieviruses (CVBs) are the human enterovirus B species of the *Picornaviridae* family. They are divided into 6 serotypes (CVB1-6) and are the major pathogens of human viral myocarditis that can lead to dilated cardiomyopathy and cardiac failure [66]. Zhong’s group determined that miR-342-5p could suppress CVB3 biogenesis by targeting its 2C-coding sequence [67]. They also observed that miR-10a* upregulated CVB3 biosynthesis by targeting the 3D-coding sequence. MiR10a* was detectable in the cardiac tissue of suckling Balb/c mice, suggesting that miR10a* might affect CVB3 replication during its cardiac infection [61].

## Conclusion

During viral life cycle, enteroviruses use viral factors and multiple host factors to mediate crucial reactions during their life cycle, including receptor binding, IRES-mediated translation, viral RNA replication, and viral assembly. However, tissue-specific viral virulence remains unclear from cell-based system to animal model, and requires further investigation in the future. Small RNAs encoded by viruses or hosts might play vital roles in complex signaling pathways of the virus-host interaction network; this is also a critical process requiring further investigation.

## Competing interests

The authors declare that they have no competing interests.

## Authors’ contributions

JYL wrote the manuscript; SRS critically revised the manuscript. Both authors have read and approved the final manuscript.
